# Matrine Protects Cardiomyocytes Against Hyperglycemic Stress by Promoting Mitofusin 2-Induced Mitochondrial Fusion

This article has been retracted.

**DOI:** 10.3389/fphys.2020.597429

**Published:** 2021-02-03

**Authors:** Tong Xiao, Jie Huang, Yuan Liu, Yujie Zhao, Manman Wei

**Affiliations:** ^1^Endocrinology and Geriatric Department, Henan Provincial Chest Hospital, Zhengzhou, China; ^2^Department of Ultrasonography, Affiliated Tumor Hospital of Zhengzhou University (Henan Cancer Hospital), Zhengzhou, China; ^3^Department of Cardiovascular, Henan Provincial Chest Hospital, Zhengzhou, China

**Keywords:** matrine, mitochondrial fusion, Mfn2, cardiomyocyte, oxidative stress, apoptosis

## Abstract

Matrine, an active component of *Sophora flavescens* Ait root extracts, has been used in China for years to treat cancer and viral hepatitis. In the present study, we explored the effects of matrine on hyperglycemia-treated cardiomyocytes. Cardiomyocyte function, oxidative stress, cellular viability, and mitochondrial fusion were assessed through immunofluorescence, quantitative real-time PCR (qRT-PCR), enzyme-linked immunosorbent assays, and RNA interference. Matrine treatment suppressed hyperglycemia-induced oxidative stress in cardiomyocytes by upregulating transcription of nuclear factor erythroid 2-like 2 and heme oxygenase-1. Matrine also improved cardiomyocyte contractile and relaxation function during hyperglycemia, and it reduced hyperglycemia-induced cardiomyocyte death by inhibiting mitochondrial apoptosis. Matrine treatment increased the transcription of mitochondrial fusion-related genes and thus attenuated the proportion of fragmented mitochondria in cardiomyocytes. Inhibiting mitochondrial fusion by knocking down mitofusin 2 (Mfn2) abolished the cardioprotective effects of matrine during hyperglycemia. These results demonstrate that matrine could be an effective drug to alleviate hyperglycemia-induced cardiomyocyte damage by activating Mfn2-induced mitochondrial fusion.

## Introduction

The incidence and mortality of diabetic cardiomyopathy are still high in most countries (Makrecka-Kuka et al., 2020). Although anti-diabetic drugs such as insulin are available to control blood glucose, no significant cardiovascular benefits have been observed in patients treated with insulin (Mamet et al., 2019; Vecchie et al., 2019), and treatment strategies that both reduce hyperglycemia and attenuate cardiac damage are limited. Therefore, in-depth research is needed to determine the pathological mechanisms of myocardial injury and ventricular remodeling during chronic hyperglycemia, and to identify additional treatment targets and schemes to prevent the adverse effects of diabetic cardiomyopathy (Sun et al., 2019).

Mitochondria are networked, plastic organelles that actively undergo fusion and fission to optimize their function and quality (Li et al., 2020; Wang et al., 2020c). Mitochondrial fusion allows the contents of partially damaged mitochondria to be intermixed and exchanged, presumably to counteract the decline of mitochondrial function (Delmotte and Sieck, 2019; Hernandez-Resendiz et al., 2020). However, in diabetic cardiomyopathy, the equilibrium between mitochondrial fission and fusion is disturbed and shifted toward mitochondrial fission. This mitochondrial phenotype has been found to precede the onset of cardiac functional and structural changes in experimental models, suggesting that abnormal mitochondrial fusion directly promotes the development of diabetic cardiomyopathy (Zhou et al., 2018c,d; Lee et al., 2019). Notably, recent studies have demonstrated that mitochondrial fission contributes to the pathology of hyperglycemia-induced cardiac damage (Zhou et al., 2018c; Hu et al., 2019b). However, the influence of mitochondrial fusion on the course of diabetic cardiomyopathy has not yet been described.

Matrine is an alkaloid found in plants from the genus *Sophora* (Li et al., 2019b), and has a variety of pharmacological effects, including anti-oxidative, anti-cancer, and anti-apoptotic effects (Lin et al., 2019; Atef et al., 2020). Matrine was found to inhibit doxorubicin-induced cardiotoxicity by activating the adenosine monophosphate-activated protein kinase/uncoupling protein 1 signaling pathway (Hu et al., 2019a). Matrine also protects against calcium overload-induced myocardial damage by suppressing ryanodine receptor 2 (Wang et al., 2019), and attenuates myocardial ischemia-reperfusion injury by inducing the Janus kinase 2/signal transducer and activator of transcription 3 pathway (Guo et al., 2018). Importantly, matrine was reported to improve cardiac function in rats with diabetic cardiomyopathy by suppressing the reactive oxygen species (ROS)/toll-like receptor 4 signaling pathway (Liu et al., 2015). Thus, in the present study, we investigated whether matrine could activate mitochondrial fusion and protect cardiomyocytes from hyperglycemic stress.

## Materials and Methods

### Cardiomyocyte Culture and Treatment

Primary cultures of neonatal rat ventricular myocytes (passage 1) were incubated in Dulbecco’s modified Eagle’s medium (DMEM) supplemented with 10% fetal bovine serum, as previously described (Jin et al., 2018). After 16 h of serum starvation, the cardiomyocytes were treated with matrine (5 nM). Cardiomyocytes in the control group were cultured in 5.5 mmol/L standard glucose medium (control group), while those in the *in vitro* hyperglycemia injury model group were cultured in 25 mmol/L high-glucose DMEM for 12 h. Both types of medium were supplemented with 10% fetal bovine serum (Gibco, C11995500), 100 IU/ml penicillin and 100 μg/ml streptomycin. The cells were incubated in 95% air and 5% CO_2_ (Wang et al., 2020a).

### TUNEL Assay

Apoptotic DNA fragments in hyperglycemia-treated cardiomyocytes were processed using a terminal deoxynucleotidyl transferase dUTP nick end labeling (TUNEL) kit (11684795910, Roche, Switzerland) according to the manufacturer’s instructions. The steps were dehydration, proteinase K incubation, TUNEL solution incubation, hematoxylin counterstaining, and section sealing (Aluja et al., 2019). Cellular apoptosis was then observed under a microscope (CKX53, OLYMPUS, Japan). Five non-repetitive fields were randomly selected, and the percentage of TUNEL-positive cells was calculated (Bocci et al., 2019).

### Immunofluorescence

Immunofluorescence assays were performed as previously described (Aalto et al., 2019; Ansari et al., 2019a), with minor modifications. Samples were dewaxed using the antigen repair method (ethylenediaminetetraacetic acid: pH 9.0) and then preincubated with 5% bovine serum albumin in phosphate buffer for 30 min. The sections were then incubated with primary antibodies against TOM-20 (1:1000, Abcam, No. 232589) and troponin T (1:1000; Abcam, No. 8295) at 4°C overnight. After being washed with phosphate-buffered saline, the sections were incubated with secondary antibodies for 1 h (1:100; Zsbio, Beijing, China) (Arun et al., 2018). Finally, the sections were mounted with mounting medium containing 4′,6-diamidino-2-phenylindole (Beyotime, Shanghai, China), and photographed with an epifluorescence microscope (Nikon, Tokyo, Japan; Afonso and Spickett, 2019).

### ELISA

In homogenates from cultured cardiomyocytes with or without matrine, the activities of proteins of interest (including caspase-3 and caspase-9) were assessed using a commercially available kit per the manufacturer’s instructions (Sigma-Aldrich; Linkermann, 2019). In brief, proteins were collected from cardiomyocytes and then diluted in assay buffer and developer solution. The activities of caspase-3 and caspase-9 were determined based on the absorbance at 450 nm (Zhang et al., 2019).

### qRT-PCR Analysis

Total RNA was extracted from samples using EZ-10 Total RNA Mini-Prep Kit Reagent (Sangon Biotech, Shanghai, China; Bocci et al., 2019). UV spectrophotometry (Jinghua, Shanghai, China) was used to determine the total RNA concentration and purity. A First Strand cDNA Synthesis Kit (ABclonal, Wuhan, China) was used to synthesize first-strand cDNA. The qRT-PCR was performed on a real-time PCR System (Bio-Rad, Shanghai, China; Bacmeister et al., 2019). The 2^-*Δ*ΔCt^ method was applied to calculate the expression of each gene relative to the expression of *β-actin*. The primer sequences used for PCR were: *Mfn1* forward: 5'-CTGGAGC ACGTTCCTTCCTC-3', reverse: 5'-ACAGTGCGAAC TGCCTCTTG-3'; *Mfn2* forward: 5'-AGGCGAAACCAGGAGAGAC-3', reverse: 5'-CCTCCCCGATCAGAGTGAA-3'; *Opa1* forward: 5'-TTATAGAGCGATACAAGGGGGAG-3', reverse: 5'-CGCCGTCTGATTATCTTGATGAG-3'; *β-actin* forward: 5'-GGGAAATCGTG CG TGACATTAAGG-3', reverse: 5'-CAGGAAGGAAGGCTGGA AGAGTG-3' (Avalle et al., 2019; Cao et al., 2019; Colombo et al., 2019).

### MTT Assay

Cardiomyocyte viability was tested using an MTT kit according to the manufacturer’s instructions (C0009, Beyotime; Battelli et al., 2019). In short, cardiomyocytes (1 × 10^4^/ml) were seeded in 96-well plates. The cells were treated with 10 μl of 3-(4,5-dimethylthiazol-2-yl)-2,5-diphenyltetrazolium bromide (MTT) solution and cultured for 4 h. Next, 100 μl of formazan lysis solution was added to the cells and mixed appropriately, and the cells were incubated until the formazan was completely dissolved. Finally, the absorbance was measured at 570 nm on a microplate reader (24072800, Thermo Fisher, United States). The experiment was repeated three times independently (Bao et al., 2018).

### ROS and Mitochondrial Membrane Potential Detection

Reactive oxygen species (ROS) levels and the mitochondrial membrane potential in cardiomyocytes were assessed according to the specifications of an ROS detection kit (Beyotime, S0033; Darden et al., 2019) and a mitochondrial membrane potential detection kit (Solarbio, CA1310), respectively (Zhou et al., 2018b). For the determination of intracellular ROS levels, 1 × 10^5^ cardiomyocytes/well were cultured under normal conditions (control group) and then incubated with 2′,7′-dichlorodihydrofluorescein diacetate solution at 37°C for 20 min. Mitochondrial ROS levels were measured using MitoSOX staining. For the measurement of the mitochondrial membrane potential, cells were treated as described above and then incubated with 5,5′,6,6′-tetrachloro-1,1′,3,3′-tetraethyl-imidacarbocyanine (JC-1) staining solution (5 mg/ml) at 37°C for 20 min. The cells were then washed twice with JC-1 staining buffer and detected on a fluorescence microscope (Olympus FV3000RS). Fluorescence was measured at excitation/emission wavelengths of 485/580 nm (red) and then at excitation/emission wavelengths of 485/530 nm (green). The results were analyzed with Image-Pro Plus software.

### Statistical Analysis

Data are expressed as the mean ± SEM. When appropriate, a two-tailed Student’s *t*-test was used to compare the mean values in two groups. One-way or two-way ANOVA with Bonferroni correction was used to compare multiple means. *p* < 0.05 was considered statistically significant. Data were analyzed using GraphPad Prism (GraphPad Software, San Diego, CA, United States).

## Results

### Matrine Attenuates Hyperglycemia-Induced Oxidative Stress in Cardiomyocytes

Previous studies have suggested that oxidative stress is the primary pathological response to hyperglycemia treatment in cells (Luo et al., 2020; Zhou and Toan, 2020). Thus, we subjected cardiomyocytes to hyperglycemia with or without matrine pretreatment, and used immunofluorescence to measure intracellular and mitochondrial ROS levels. Cells in normal-glucose medium were used as the control group. As shown in Figures 1A,B, the intracellular ROS content was significantly greater in the high-glucose group than in the control group; however, matrine pretreatment reversed this increase in hyperglycemia-treated cells. Hyperglycemia treatment also increased mitochondrial ROS levels, while matrine reduced them (Figures 1C,D). These results indicated that matrine attenuated hyperglycemia-induced oxidative stress in cardiomyocytes.

**Figure 1:** Matrine attenuates hyperglycemia-induced oxidative stress in cardiomyocytes. **(A,B)** Intracellular reactive oxygen species (ROS) levels were determined using 2',7'-dichlorodihydrofluorescein diacetate. Cardiomyocytes were treated with matrine under hyperglycemic conditions. **(C,D)** Mitochondrial ROS levels were measured through MitoSOX staining. **(E–I)** Quantitative real-time PCR (qRT-PCR) was performed to evaluate the transcription of glutathione (*GSH*), superoxide dismutase (*SOD*), glutathione peroxidase (*GPX*), nuclear factor erythroid 2-like 2 (*Nrf2*), and heme oxygenase-1 (*HO-1*). H9C2 cells were treated with matrine under hyperglycemic conditions. ^*^p < 0.05.

Matrine has been reported to activate the cellular anti-oxidative system (Hu et al., 2019a). Thus, we performed quantitative real-time PCR (qRT-PCR) to evaluate the transcription of anti-oxidative genes in cardiomyocytes. As shown in Figures 1E–I, the mRNA levels of anti-oxidative genes were significantly lower in the hyperglycemia group than in the control group. Matrine treatment significantly upregulated anti-oxidative genes such as glutathione (*GSH*), superoxide dismutase (*SOD*), and glutathione peroxidase (*GPX*) in cardiomyocytes. Matrine also increased the mRNA levels of nuclear factor erythroid 2-like 2 (*Nrf2*) and heme oxygenase-1 (*HO-1*), two key proteins that maintain cellular redox balance, in hyperglycemia-treated cardiomyocytes (Figures 1E–I). These results further demonstrated that matrine alleviated hyperglycemia-induced oxidative stress in cardiomyocytes.

### Matrine Treatment Reduces Hyperglycemia-Induced Cardiomyocyte Dysfunction

Next, we examined the effects of matrine on cardiomyocyte function under hyperglycemic conditions. First, we analyzed cardiomyocyte contractility and relaxation by measuring the maximal velocities of shortening and lengthening. As shown in Figures 2A,B, the maximal velocities of shortening and lengthening were significantly lower in the hyperglycemia group than in the control group; however, matrine pretreatment ameliorated this effect. At the molecular level, a sufficient adenosine triphosphate (ATP) supply is vital for cardiomyocyte contractility and relaxation. Interestingly, intracellular ATP levels were rapidly downregulated in response to hyperglycemia treatment, but were restored by matrine supplementation in cardiomyocytes (Figure 2C).

**Figure 2:** Matrine treatment reduces hyperglycemia-induced cardiomyocyte dysfunction. **(A,B)** The maximal velocities of the shortening and lengthening rates of cardiomyocytes were determined. At least 100 cardiomyocytes were recorded. **(C)**. An ELISA was used to measure adenosine triphosphate (ATP) production in cardiomyocytes. **(D,E)** The expression of troponin T was detected through immunofluorescence. ^*^p < 0.05.

Troponin T has been identified as a critical contractile structure for the maintenance of cardiomyocyte contractility/relaxation. Hyperglycemia significantly reduced troponin T levels, while matrine reversed this change in cardiomyocytes (Figures 2D,E). These results suggested that matrine treatment reduced hyperglycemia-induced cardiomyocyte dysfunction by sustaining troponin T expression.

### Matrine Treatment Attenuates Hyperglycemia-Induced Cardiomyocyte Death by Inhibiting the Caspase-9/Caspase-3 Pathways

Irreparable cardiomyocyte damage can induce cell death and thus reduce the number of functional cardiomyocytes (Zhou et al., 2018a). Chronic cardiomyocyte death is prominent in the progression of diabetic cardiomyopathy (Yu et al., 2019). Thus, we examined the effects of matrine on hyperglycemia-induced cardiomyocyte death. First, we performed a MTT assay to analyze cardiomyocyte viability, and found that matrine pretreatment maintained cardiomyocyte viability under hyperglycemic stress (Figure 3A). Further, a TUNEL assay demonstrated that hyperglycemia increased the number of dead cardiomyocytes, while matrine treatment reduced this number to a near-normal level (Figures 3B,C), suggesting that matrine promoted the survival of hyperglycemia-treated cardiomyocytes.

**Figure 3:** Matrine treatment attenuates hyperglycemia-induced cardiomyocyte death by inhibiting the caspase-9/caspase-3 pathways. (**A)**. An 3-(4,5-dimethylthiazol-2-yl)-2,5-diphenyltetrazolium bromide (MTT) assay was used to determine the viability of cardiomyocytes under hyperglycemic conditions. **(B,C)** Terminal deoxynucleotidyl transferase dUTP nick end labeling (TUNEL) staining was applied to observe cell death in response to hyperglycemic stress. **(D,E)** 5,5',6,6'-tetrachloro-1,1',3,3'-tetraethyl-imidacarbocyanine (JC-1) probe was used to evaluate the mitochondrial membrane potential in cardiomyocytes under hyperglycemic conditions. **(F,G)** ELISAs were used to evaluate the activities of caspase-3 and caspase-9 in cardiomyocytes under hyperglycemic conditions. ^*^p < 0.05.

A reduced mitochondrial membrane potential has been identified as an early feature of cardiomyocyte death through mitochondrial apoptotic pathways (Dassanayaka et al., 2019; Heusch, 2019). Using immunofluorescence, we found that hyperglycemia disrupted the mitochondrial membrane potential, whereas matrine effectively sustained it in high-glucose-treated cells (Figures 3D,E). We also performed ELISAs to analyze the activity of proteins in the mitochondrial apoptotic pathway, including caspase-3 and caspase-9. As shown in Figures 3F,G, the activities of caspase-3 and caspase-9 were significantly greater in the hyperglycemia group than in the control group, but matrine prevented this alteration. These results indicated that matrine effectively alleviated hyperglycemia-induced cardiomyocyte death by inhibiting caspase-9-induced mitochondrial apoptosis.

### Matrine Activates Mitochondrial Fusion by Upregulating Mitofusin 2

To determine whether matrine enhanced cardiomyocyte viability and function by promoting mitochondrial fusion, we performed an immunofluorescence assay (Zhou et al., 2018e). As shown in Figures 4A–C, mitochondria fusion was inhibited in the hyperglycemia group compared with the control group, as evidenced by the reduced mitochondrial length and increased proportion of fragmented mitochondria in the cardiomyocytes. Matrine treatment significantly elevated the average length of the mitochondria and reduced the proportion of fragmented mitochondria (Figures 4A–C).

**Figure 4:** Matrine activates mitochondrial fusion by upregulating mitofusin 2 (*Mfn2*). **(A–C)** The mitochondrial morphology was observed through immunofluorescence staining. The proportion of fragmented mitochondria was recorded, and the average length of the mitochondria was measured. **(D–F)** The transcription of mitochondrial fusion-related genes was measured through qRT-PCR. **(G–I)** The levels of anti-fusion genes in hyperglycemia-treated cardiomyocytes were determined through qRT-PCR. ^*^p < 0.05.

To verify that matrine induced mitochondrial fusion, we assessed the mRNA levels of proteins involved in mitochondrial fusion. As shown in Figures 4D–F, the mRNA levels of *Mfn1*, mitofusin 2 (*Mfn2*), and *Opa1* were significantly lower in the hyperglycemia group than in the control group; however, matrine attenuated this reduction. We also found that hyperglycemia significantly increased the mRNA levels of anti-fusion genes in cardiomyocytes, while matrine inhibited this upregulation (Figures 4G–I). These data suggested that matrine improved mitochondrial fusion in cardiomyocytes.

### Inhibition of Mitochondrial Fusion Abolishes the Cardioprotective Effects of Matrine

Lastly, we analyzed whether mitochondrial fusion was required for the cardioprotective effects of matrine. Previous studies have indicated that mitochondrial fusion is primarily stimulated by Mfn2 (Wang et al., 2020b,d). Thus, we transfected cardiomyocytes with siRNA against *Mfn2* and measured cardiomyocyte viability. As shown in Figure 5A, although matrine sustained cardiomyocyte viability under hyperglycemic conditions, siRNA against *Mfn2* abolished this protective action. Additionally, while matrine maintained the expression of troponin T in hyperglycemia-treated cardiomyocytes, siRNA against *Mfn2* attenuated this effect (Figures 5B,C). Transfection with siRNA against *Mfn2* also repressed the anti-oxidative effects of matrine in cardiomyocytes, as evidenced by the reduced mRNA levels of *Nrf2* and *HO-1* (Figures 5D,E). These results confirmed that Mfn2-induced mitochondrial fusion was required for the cardioprotective effects of matrine under hyperglycemic conditions.

**Figure 5:** Inhibition of mitochondrial fusion abolishes the cardioprotective effects of matrine. (**A)**. Cardiomyocytes were transfected with siRNA against *Mfn2* before being treated with matrine under hyperglycemic conditions. Then, cell viability was determined through an MTT assay. **(B,C)** The expression of troponin T was determined through an immunofluorescence assay. **(D,E)** RNA was isolated from cardiomyocytes transfected with *Mfn2* siRNA, and then the mRNA levels of *Nrf2* and *HO-1* were determined through qRT-PCR. ^*^p < 0.05.

## Discussion

The uncontrolled spread of type 2 diabetes mellitus is primarily due to delays in proper diagnosis and illiteracy regarding diabetes management. It is estimated that around 592 million people will have diabetes by 2035 (Li et al., 2019a). In 2014, around 4.9 million deaths due to diabetes were reported (DeLeon-Pennell et al., 2018). Thus, there is a great need to develop new anti-diabetic treatments and modify the existing therapeutic approaches (Sowton et al., 2019) in order to attenuate the complications of diabetes, especially microvascular complications (retinopathy, nephropathy, and neuropathy), macrovascular complications (ischemic heart disease, stroke, and peripheral vascular disease), and the diminished quality of life (Heusch, 2018; Karwi et al., 2018).

Clinical data have demonstrated that there is a bidirectional relationship between diabetes mellitus and cardiovascular diseases, as well as heart failure (Song et al., 2018). Various factors associated with diabetes mellitus, such as impaired calcium homeostasis, altered free fatty acid metabolism, an unbalanced redox state, and increased advanced glycation end products, contribute to cardiovascular complications (Riehle and Bauersachs, 2018; Zhang et al., 2018; Zheng et al., 2018). On the other hand, hypoperfusion of the liver and pancreas, treatment with *β*-blockers and diuretics, and dysfunction of the autonomic nervous system due to heart failure can impair glucose metabolism (Ansari et al., 2019b). During anti-diabetic drug discovery, targeting common molecules between diabetes mellitus and cardiovascular diseases [such as peroxisome proliferator-activated receptors (PPARs), which are involved in insulin resistance, glucose and lipid metabolism, and systolic or diastolic activity of the left ventricle] may provide a solution to these reciprocal complications (Wu et al., 2018). Preclinical studies have demonstrated that PPAR activation can upregulate fatty acid oxidation genes, improve ventricular contraction, and reduce cardiac remodeling *via* anti-inflammatory, anti-oxidant, anti-fibrotic, and anti-apoptotic mechanisms (Kanwal et al., 2019). Our data indicated that matrine, an alkaloid found in plants from the genus *Sophora*, can be used to prevent or attenuate the effects of hyperglycemia on cardiomyocytes. This therapeutic approach may have cardiovascular benefits for patients with diabetes; however, we have not tested the safety and effectiveness of insulin and matrine in combination, so this point requires further exploration.

The currently available therapeutics does not address the high mortality rate of diabetes mellitus patients due to cardiac dysfunction (Eid et al., 2018; Knapp et al., 2019). While the existing anti-diabetic medications can restrain increasing blood glucose levels, their adverse side effects and the complications associated with diabetes demonstrate the need to develop better drugs (Gaspar et al., 2018). The molecular mechanisms of cardiomyocyte damage in diabetes are not fully understood. Although mitochondrial fission has been reported as an independent risk factor for the development of cardiomyocyte dysfunction (Choi et al., 2016; Fang et al., 2018), the influence of mitochondrial fusion on hyperglycemia-treated cardiomyocytes has not been clarified. Our cellular experiments revealed that the activation of mitochondrial fusion had cardioprotective effects. By promoting mitochondrial fusion, matrine attenuated hyperglycemia-induced oxidative stress, contractile/relaxation dysfunction, and mitochondrial apoptosis in cardiomyocytes. In contrast, inhibiting mitochondrial fusion using siRNA against *Mfn2* re-induced redox imbalance, cardiomyocyte dysfunction, and death in matrine-treated cells. These findings illustrated the importance of mitochondrial fusion for cardioprotection.

The benefits of Mfn2 in cardiovascular disorders have been reported recently. For example, the activation of mitochondrial fusion was found to enhance myocardial resistance to ischemia-reperfusion injury (Wang et al., 2020f). Overexpression of *Mfn1* upregulated mitochondrial fusion, protecting the heart against hypertrophy by circumventing the miR-153-3p signaling pathway (Wang et al., 2020g). Although enhancing mitochondrial dynamics has been reported as a therapeutic intervention in diabetic cardiomyopathy, most studies have focused on the effects of mitochondrial fission and mitophagy on mitochondrial homeostasis (Zhou et al., 2019; Wang et al., 2020e). Our data have provided novel insights into the molecular mechanisms by which mitochondrial fusion exerts cardioprotective effects.

In conclusion, we have demonstrated that matrine may be an effective drug to attenuate hyperglycemia-induced cardiomyocyte damage. Matrine supplementation upregulated *Mfn2* expression and thus activated mitochondrial fusion, protecting cardiomyocytes from oxidative stress and apoptosis. Clinical data would be useful to support our findings.

## Data Availability Statement

The original contributions presented in the study are included in the article/supplementary material, further inquiries can be directed to the corresponding author.

## Author Contributions

MW, TX, and JH designed and performed the experiments. YL and YZ collected the data and prepared figures and/or tables. All authors contributed to the article and approved the submitted version.

### Conflict of Interest

The authors declare that the research was conducted in the absence of any commercial or financial relationships that could be construed as a potential conflict of interest.

## References

[ref1] AaltoA. L.MohanA. K.SchwintzerL.KupkaS.KietzC.WalczakH.. (2019). M1-linked ubiquitination by LUBEL is required for inflammatory responses to oral infection in *Drosophila*. Cell Death Differ. 26, 860–876. 10.1038/s41418-018-0164-x, PMID: 30026495PMC6462001

[ref2] AfonsoC. B.SpickettC. M. (2019). Lipoproteins as targets and markers of lipoxidation. Redox Biol. 23:101066. 10.1016/j.redox.2018.101066, PMID: 30579928PMC6859580

[ref3] AlujaD.InserteJ.PenelaP.RamosP.RibasC.IniguezM. A.. (2019). Calpains mediate isoproterenol-induced hypertrophy through modulation of GRK2. Basic Res. Cardiol. 114:21. 10.1007/s00395-019-0730-5, PMID: 30915659

[ref4] AnsariM.GopalakrishnanS.KurianG. A. (2019b). Streptozotocin-induced type II diabetic rat administered with nonobesogenic high-fat diet is highly susceptible to myocardial ischemia-reperfusion injury: an insight into the function of mitochondria. J. Cell. Physiol. 234, 4104–4114. 10.1002/jcp.27217, PMID: 30191974

[ref5] AnsariD.TorenW.ZhouQ.HuD.AnderssonR. (2019a). Proteomic and genomic profiling of pancreatic cancer. Cell Biol. Toxicol. 35, 333–343. 10.1007/s10565-019-09465-9, PMID: 30771135PMC6757097

[ref6] ArunK. G.SharanyaC. S.SadasivanC. (2018). Computational and experimental validation of morin as adenosine deaminase inhibitor. J. Recept. Signal Transduct. Res. 38, 240–245. 10.1080/10799893.2018.1476543, PMID: 29843562

[ref7] AtefM. M.El-DeebO. S.SadekM. T.Abo El GheitR. E.EmamM. N.HafezY. M.. (2020). Targeting ERK/COX-2 signaling pathway in permethrin-induced testicular toxicity: a possible modulating effect of matrine. Mol. Biol. Rep. 47, 247–259. 10.1007/s11033-019-05125-7, PMID: 31621018

[ref8] AvalleL.CamporealeA.MorcianoG.CarocciaN.GhettiE.OrecchiaV.. (2019). STAT3 localizes to the ER, acting as a gatekeeper for ER-mitochondrion Ca(2+) fluxes and apoptotic responses. Cell Death Differ. 26, 932–942. 10.1038/s41418-018-0171-y, PMID: 30042492PMC6214529

[ref9] BacmeisterL.SchwarzlM.WarnkeS.StoffersB.BlankenbergS.WestermannD.. (2019). Inflammation and fibrosis in murine models of heart failure. Basic Res. Cardiol. 114:19. 10.1007/s00395-019-0722-5, PMID: 30887214

[ref10] BaoY.ZhouL.DaiD.ZhuX.HuY.QiuY. (2018). Discover potential inhibitors for PFKFB3 using 3D-QSAR, virtual screening, molecular docking and molecular dynamics simulation. J. Recept. Signal Transduct. Res. 38, 413–431. 10.1080/10799893.2018.1564150, PMID: 30822195

[ref11] BattelliM. G.BortolottiM.PolitoL.BolognesiA. (2019). Metabolic syndrome and cancer risk: the role of xanthine oxidoreductase. Redox Biol. 21:101070. 10.1016/j.redox.2018.101070, PMID: 30576922PMC6302121

[ref12] BocciM.SjolundJ.KurzejamskaE.LindgrenD.MarzoukaN. A.BartoschekM.. (2019). Activin receptor-like kinase 1 is associated with immune cell infiltration and regulates CLEC14A transcription in cancer. Angiogenesis 22, 117–131. 10.1007/s10456-018-9642-5, PMID: 30132150PMC6510886

[ref13] CaoX.HuY.LuoS.WangY.GongT.SunX.. (2019). Neutrophil-mimicking therapeutic nanoparticles for targeted chemotherapy of pancreatic carcinoma. Acta Pharm. Sin. B 9, 575–589. 10.1016/j.apsb.2018.12.009, PMID: 31193785PMC6543032

[ref14] ChoiH. Y.ParkJ. H.JangW. B.JiS. T.JungS. Y.KimD. Y.. (2016). High glucose causes human cardiac progenitor cell dysfunction by promoting mitochondrial fission: role of a GLUT1 blocker. Biomol. Ther. 24, 363–370. 10.4062/biomolther.2016.097, PMID: 27350339PMC4930279

[ref15] ColomboG.GaravagliaM. L.AstoriE.GiustariniD.RossiR.MilzaniA.. (2019). Protein carbonylation in human bronchial epithelial cells exposed to cigarette smoke extract. Cell Biol. Toxicol. 35, 345–360. 10.1007/s10565-019-09460-0, PMID: 30648195

[ref16] DardenJ.PayneL. B.ZhaoH.ChappellJ. C. (2019). Excess vascular endothelial growth factor-A disrupts pericyte recruitment during blood vessel formation. Angiogenesis 22, 167–183. 10.1007/s10456-018-9648-z, PMID: 30238211PMC6360133

[ref17] DassanayakaS.BrittianK. R.JurkovicA.HigginsL. A.AudamT. N.LongB. W.. (2019). E2f1 deletion attenuates infarct-induced ventricular remodeling without affecting O-GlcNAcylation. Basic Res. Cardiol. 114:28. 10.1007/s00395-019-0737-y, PMID: 31152247PMC7278029

[ref18] DeLeon-PennellK. Y.MoutonA. J.EroO. K.MaY.IyerR. P.FlynnE. R.. (2018). LXR/RXR signaling and neutrophil phenotype following myocardial infarction classify sex differences in remodeling. Basic Res. Cardiol. 113:40. 10.1007/s00395-018-0699-5, PMID: 30132266PMC6105266

[ref19] DelmotteP.SieckG. C. (2019). Endoplasmic reticulum stress and mitochondrial function in airway smooth muscle. Front. Cell Dev. Biol. 7:374. 10.3389/fcell.2019.00374, PMID: 32010691PMC6974519

[ref20] EidR. A.AlkhateebM. A.EleawaS.Al-HashemF. H.Al-ShraimM.El-KottA. F.. (2018). Cardioprotective effect of ghrelin against myocardial infarction-induced left ventricular injury via inhibition of SOCS3 and activation of JAK2/STAT3 signaling. Basic Res. Cardiol. 113:13. 10.1007/s00395-018-0671-4, PMID: 29392420

[ref21] FangW. J.WangC. J.HeY.ZhouY. L.PengX. D.LiuS. K. (2018). Resveratrol alleviates diabetic cardiomyopathy in rats by improving mitochondrial function through PGC-1alpha deacetylation. Acta Pharmacol. Sin. 39, 59–73. 10.1038/aps.2017.50, PMID: 28770830PMC5758665

[ref22] GasparA.LourencoA. P.PereiraM. A.AzevedoP.Roncon-AlbuquerqueR.Jr.MarquesJ.. (2018). Randomized controlled trial of remote ischaemic conditioning in ST-elevation myocardial infarction as adjuvant to primary angioplasty (RIC-STEMI). Basic Res. Cardiol. 113:14. 10.1007/s00395-018-0672-3, PMID: 29516192

[ref23] GuoS.GaoC.XiaoW.ZhangJ.QuY.LiJ.. (2018). Matrine protects cardiomyocytes from ischemia/reperfusion injury by regulating HSP70 expression via activation of the JAK2/STAT3 pathway. Shock 50, 664–670. 10.1097/SHK.0000000000001108, PMID: 29394239

[ref24] Hernandez-ResendizS.PrunierF.GiraoH.DornG.HausenloyD. J.ActionE. -C. C. (2020). Targeting mitochondrial fusion and fission proteins for cardioprotection. J. Cell. Mol. Med. 24, 6571–6585. 10.1111/jcmm.15384, PMID: 32406208PMC7299693

[ref25] HeuschG. (2018). 25 years of remote ischemic conditioning: from laboratory curiosity to clinical outcome. Basic Res. Cardiol. 113:15. 10.1007/s00395-018-0673-2, PMID: 29516255

[ref26] HeuschG. (2019). Coronary microvascular obstruction: the new frontier in cardioprotection. Basic Res. Cardiol. 114:45. 10.1007/s00395-019-0756-8, PMID: 31617010

[ref27] HuL.DingM.TangD.GaoE.LiC.WangK.. (2019b). Targeting mitochondrial dynamics by regulating Mfn2 for therapeutic intervention in diabetic cardiomyopathy. Theranostics 9, 3687–3706. 10.7150/thno.33684, PMID: 31281507PMC6587356

[ref28] HuC.ZhangX.WeiW.ZhangN.WuH.MaZ.. (2019a). Matrine attenuates oxidative stress and cardiomyocyte apoptosis in doxorubicin-induced cardiotoxicity via maintaining AMPKalpha/UCP2 pathway. Acta Pharm. Sin. B 9, 690–701. 10.1016/j.apsb.2019.03.003, PMID: 31384530PMC6664099

[ref29] JinQ.LiR.HuN.XinT.ZhuP.HuS.. (2018). DUSP1 alleviates cardiac ischemia/reperfusion injury by suppressing the Mff-required mitochondrial fission and Bnip3-related mitophagy via the JNK pathways. Redox Biol. 14, 576–587. 10.1016/j.redox.2017.11.004, PMID: 29149759PMC5691221

[ref30] KanwalA.PillaiV. B.SamantS.GuptaM.GuptaM. P. (2019). The nuclear and mitochondrial sirtuins, Sirt6 and Sirt3, regulate each other's activity and protect the heart from developing obesity-mediated diabetic cardiomyopathy. FASEB J. 33, 10872–10888. 10.1096/fj.201900767R, PMID: 31318577PMC6766651

[ref31] KarwiQ. G.BiceJ. S.BaxterG. F. (2018). Pre- and postconditioning the heart with hydrogen sulfide (H2S) against ischemia/reperfusion injury in vivo: a systematic review and meta-analysis. Basic Res. Cardiol. 113:6. 10.1007/s00395-017-0664-8, PMID: 29242986PMC5730622

[ref32] KnappM.TuX.WuR. (2019). Vascular endothelial dysfunction, a major mediator in diabetic cardiomyopathy. Acta Pharmacol. Sin. 40, 1–8. 10.1038/s41401-018-0042-6, PMID: 29867137PMC6318313

[ref33] LeeT. W.KaoY. H.ChenY. J.ChaoT. F.LeeT. I. (2019). Therapeutic potential of vitamin D in AGE/RAGE-related cardiovascular diseases. Cell. Mol. Life Sci. 76, 4103–4115. 10.1007/s00018-019-03204-3, PMID: 31250032PMC11105755

[ref34] LiH.DaiB.FanJ.ChenC.NieX.YinZ.. (2019a). The different roles of miRNA-92a-2-5p and let-7b-5p in mitochondrial translation in db/db mice. Mol. Ther. Nucleic Acids 17, 424–435. 10.1016/j.omtn.2019.06.013, PMID: 31319246PMC6637210

[ref35] LiR. B.ToanS.ZhouH. (2020). Role of mitochondrial quality control in the pathogenesis of nonalcoholic fatty liver disease. Aging 12, 6467–6485. 10.18632/aging.102972, PMID: 32213662PMC7185127

[ref36] LiW.WangH.DongA. (2019b). Preparative separation of alkaloids from stem of euchresta tubulosa dunn. by high-speed counter-current chromatography using stepwise elution. Molecules 24:4602. 10.3390/molecules24244602, PMID: 31888219PMC6943640

[ref37] LinG.WuY.CaiF.LiZ.SuS.WangJ.. (2019). Matrine promotes human myeloid leukemia cells apoptosis through warburg effect mediated by hexokinase 2. Front. Pharmacol. 10:1069. 10.3389/fphar.2019.01069, PMID: 31607919PMC6771294

[ref38] LinkermannA. (2019). Death and fire-the concept of necroinflammation. Cell Death Differ. 26, 1–3. 10.1038/s41418-018-0218-0, PMID: 30470796PMC6294805

[ref39] LiuZ. W.WangJ. K.QiuC.GuanG. C.LiuX. H.LiS. J.. (2015). Matrine pretreatment improves cardiac function in rats with diabetic cardiomyopathy via suppressing ROS/TLR-4 signaling pathway. Acta Pharmacol. Sin. 36, 323–333. 10.1038/aps.2014.127, PMID: 25619390PMC4349921

[ref40] LuoJ.YanD.LiS.LiuS.ZengF.CheungC. W.. (2020). Allopurinol reduces oxidative stress and activates Nrf2/p62 to attenuate diabetic cardiomyopathy in rats. J. Cell. Mol. Med. 24, 1760–1773. 10.1111/jcmm.14870, PMID: 31856386PMC6991641

[ref41] Makrecka-KukaM.LiepinshE.MurrayA. J.LemieuxH.DambrovaM.TeppK.. (2020). Altered mitochondrial metabolism in the insulin-resistant heart. Acta Physiol. 228:e13430. 10.1111/apha.13430, PMID: 31840389

[ref42] MametH.PetrieM. C.RocchiccioliP. (2019). Type 1 diabetes mellitus and coronary revascularization. Cardiovasc. Endocrinol. Metab. 8, 35–38. 10.1097/XCE.0000000000000166, PMID: 31646296PMC6739890

[ref43] RiehleC.BauersachsJ. (2018). Of mice and men: models and mechanisms of diabetic cardiomyopathy. Basic Res. Cardiol. 114:2. 10.1007/s00395-018-0711-0, PMID: 30443826PMC6244639

[ref44] SongJ.YangR.YangJ.ZhouL. (2018). Mitochondrial dysfunction-associated arrhythmogenic substrates in diabetes mellitus. Front. Physiol. 9:1670. 10.3389/fphys.2018.01670, PMID: 30574091PMC6291470

[ref45] SowtonA. P.GriffinJ. L.MurrayA. J. (2019). Metabolic profiling of the diabetic heart: toward a richer picture. Front. Physiol. 10:639. 10.3389/fphys.2019.00639, PMID: 31214041PMC6555155

[ref46] SunL.YuM.ZhouT.ZhangS.HeG.WangG.. (2019). Current advances in the study of diabetic cardiomyopathy: from clinicopathological features to molecular therapeutics (review). Mol. Med. Rep. 20, 2051–2062. 10.3892/mmr.2019.10473, PMID: 31322242

[ref47] VecchieA.MontecuccoF.CarboneF.DallegriF.BonaventuraA. (2019). Diabetes and vascular disease: is it all about glycemia? Curr. Pharm. Des. 25, 3112–3127. 10.2174/1381612825666190830181944, PMID: 31470783

[ref48] WangK.LiuZ.ZhaoM.ZhangF.WangK.FengN.. (2020f). Kappa-opioid receptor activation promotes mitochondrial fusion and enhances myocardial resistance to ischemia and reperfusion injury via STAT3-OPA1 pathway. Eur. J. Pharmacol. 874:172987. 10.1016/j.ejphar.2020.172987, PMID: 32032598

[ref49] WangJ.TangZ.ZhangY.QiuC.ZhuL.ZhaoN.. (2019). Matrine alleviates AGEs-induced cardiac dysfunctions by attenuating calcium overload via reducing ryanodine receptor 2 activity. Eur. J. Pharmacol. 842, 118–124. 10.1016/j.ejphar.2018.10.010, PMID: 30339815

[ref50] WangJ.ToanS.LiR.ZhouH. (2020a). Melatonin fine-tunes intracellular calcium signals and eliminates myocardial damage through the IP3R/MCU pathways in cardiorenal syndrome type 3. Biochem. Pharmacol. 174:113832. 10.1016/j.bcp.2020.113832, PMID: 32006470

[ref51] WangJ.ToanS.ZhouH. (2020b). Mitochondrial quality control in cardiac microvascular ischemia-reperfusion injury: new insights into the mechanisms and therapeutic potentials. Pharmacol. Res. 156:104771. 10.1016/j.phrs.2020.104771, PMID: 32234339

[ref52] WangJ.ToanS.ZhouH. (2020c). New insights into the role of mitochondria in cardiac microvascular ischemia/reperfusion injury. Angiogenesis 23, 299–314. 10.1007/s10456-020-09720-2, PMID: 32246225

[ref53] WangT.ZhaiM.XuS.PonnusamyM.HuangY.LiuC. Y.. (2020g). NFATc3-dependent expression of miR-153-3p promotes mitochondrial fragmentation in cardiac hypertrophy by impairing mitofusin-1 expression. Theranostics 10, 553–566. 10.7150/thno.37181, PMID: 31903137PMC6929994

[ref54] WangJ.ZhuP.LiR.RenJ.ZhangY.ZhouH. (2020d). Bax inhibitor 1 preserves mitochondrial homeostasis in acute kidney injury through promoting mitochondrial retention of PHB2. Theranostics 10, 384–397. 10.7150/thno.40098, PMID: 31903127PMC6929616

[ref55] WangJ.ZhuP.LiR.RenJ.ZhouH. (2020e). Fundc1-dependent mitophagy is obligatory to ischemic preconditioning-conferred renoprotection in ischemic AKI via suppression of Drp1-mediated mitochondrial fission. Redox Biol. 30:101415. 10.1016/j.redox.2019.101415, PMID: 31901590PMC6940662

[ref56] WuM.YangY.WangM.ZengF.LiQ.LiuW.. (2018). Exogenous pancreatic kallikrein improves diabetic cardiomyopathy in streptozotocin-induced diabetes. Front. Pharmacol. 9:855. 10.3389/fphar.2018.00855, PMID: 30131697PMC6091235

[ref57] YuX.SeowH. J.WangH.AnthonyD.BozinovskiS.LinL.. (2019). Matrine reduces cigarette smoke-induced airway neutrophilic inflammation by enhancing neutrophil apoptosis. Clin. Sci. 133, 551–564. 10.1042/CS20180912, PMID: 30733313

[ref58] ZhangH.JinB.FaberJ. E. (2019). Mouse models of Alzheimer's disease cause rarefaction of pial collaterals and increased severity of ischemic stroke. Angiogenesis 22, 263–279. 10.1007/s10456-018-9655-0, PMID: 30519973PMC6475514

[ref59] ZhangB.ZhangJ.ZhangC.ZhangX.YeJ.KuangS.. (2018). Notoginsenoside R1 protects against diabetic cardiomyopathy through activating estrogen receptor alpha and its downstream signaling. Front. Pharmacol. 9:1227. 10.3389/fphar.2018.01227, PMID: 30450046PMC6224485

[ref60] ZhengJ.ChengJ.ZhengS.ZhangL.GuoX.ZhangJ.. (2018). Physical exercise and its protective effects on diabetic cardiomyopathy: what is the evidence? Front. Endocrinol. 9:729. 10.3389/fendo.2018.00729, PMID: 30559720PMC6286969

[ref61] ZhouH.ShiC.HuS.ZhuH.RenJ.ChenY. (2018a). BI1 is associated with microvascular protection in cardiac ischemia reperfusion injury via repressing Syk-Nox2-Drp1-mitochondrial fission pathways. Angiogenesis 21, 599–615. 10.1007/s10456-018-9611-z, PMID: 29623489

[ref62] ZhouH.ToanS. (2020). Pathological roles of mitochondrial oxidative stress and mitochondrial dynamics in cardiac microvascular ischemia/reperfusion injury. Biomolecules 10:85. 10.3390/biom10010085, PMID: 31948043PMC7023463

[ref63] ZhouH.WangS.ZhuP.HuS.ChenY.RenJ. (2018c). Empagliflozin rescues diabetic myocardial microvascular injury via AMPK-mediated inhibition of mitochondrial fission. Redox Biol. 15, 335–346. 10.1016/j.redox.2017.12.019, PMID: 29306791PMC5756062

[ref64] ZhouH.WangJ.ZhuP.ZhuH.ToanS.HuS.. (2018b). NR4A1 aggravates the cardiac microvascular ischemia reperfusion injury through suppressing FUNDC1-mediated mitophagy and promoting Mff-required mitochondrial fission by CK2alpha. Basic Res. Cardiol. 113:23. 10.1007/s00395-018-0682-1, PMID: 29744594

[ref65] ZhouH.YueY.WangJ.MaQ.ChenY. (2018d). Melatonin therapy for diabetic cardiomyopathy: a mechanism involving Syk-mitochondrial complex I-SERCA pathway. Cell. Signal. 47, 88–100. 10.1016/j.cellsig.2018.03.012, PMID: 29601906

[ref66] ZhouH.ZhuP.WangJ.ToanS.RenJ. (2019). DNA-PKcs promotes alcohol-related liver disease by activating Drp1-related mitochondrial fission and repressing FUNDC1-required mitophagy. Signal Transduct. Target. Ther. 4:56. 10.1038/s41392-019-0094-1, PMID: 31839999PMC6895206

[ref67] ZhouH.ZhuP.WangJ.ZhuH.RenJ.ChenY. (2018e). Pathogenesis of cardiac ischemia reperfusion injury is associated with CK2alpha-disturbed mitochondrial homeostasis via suppression of FUNDC1-related mitophagy. Cell Death Differ. 25, 1080–1093. 10.1038/s41418-018-0086-7, PMID: 29540794PMC5988750

